The article "Targeting the lncRNA FGD5-AS1/miR-497-5p/PD-L1 Axis Inhibits Malignant Phenotypes in Colon Cancer (CC)" was retracted in 2023. Reasons: signs of a paper mill; suspected computer-generated content; unreliable results or conclusions; concerns about the data.

# Targeting the lncRNA FGD5-AS1/miR-497-5p/PD-L1 Axis Inhibits Malignant Phenotypes in Colon Cancer (CC)

**DOI:** 10.1155/2022/1133332

**Published:** 2022-07-06

**Authors:** Lijuan Zhang, Xinyi Cai, Youguo Dai, Yun Chen, Jing Yu, Yongchun Zhou

**Affiliations:** ^1^The Department of Pathology, The Third Affiliated Hospital of Kunming Medical University (Yunnan Cancer Hospital), Kunzhou Road No. 519, Kunming City, 650100 Yunnan Province, China; ^2^The Department of Colorectal Surgery, The Third Affiliated Hospital of Kunming Medical University (Yunnan Cancer Hospital), Kunzhou Road No. 519, Kunming City, 650100 Yunnan Province, China; ^3^The Department of Gastroenterology, The Third Affiliated Hospital of Kunming Medical University (Yunnan Cancer Hospital), Kunzhou Road No. 519, Kunming City, 650100 Yunnan Province, China; ^4^The Department of Gynecology, The Third Affiliated Hospital of Kunming Medical University (Yunnan Cancer Hospital), Kunzhou Road No. 519, Kunming City, 650100 Yunnan Province, China; ^5^Molecular Diagnosis Center of Yunnan Cancer Center, The Third Affiliated Hospital of Kunming Medical University (Yunnan Cancer Hospital), Kunzhou Road No. 519, Kunming City, 650100 Yunnan Province, China

## Abstract

Long noncoding RNAs (lncRNAs) regulate cancer progression and drug resistance. However, the role of lncRNA FGD5-AS1 in regulating colon cancer (CC) progression is still largely unknown. Hence, this study investigated the role of lncRNA FGD5-AS1 in regulating colon cancer (CC) progression and found that lncRNA FGD5-AS1 regulated miR-497-5p/PD-L1 axis to promote cancer progression in CC cells *in vitro* and *in vivo*. Specifically, we found that lncRNA FGD5-AS1 and PD-L1 tended to be high-expressed, while miR-497-5p was low-expressed in CC tissues and cell lines compared to the normal adjacent tissues and cells. Next, we found that lncRNA FGD5-AS1 positively regulated PD-L1 in CC cells by sponging miR-497-5p. Finally, our gain- and loss-of-function experiments evidenced that the lncRNA FGD5-AS1/miR-497-5p/PD-L1 axis regulates CC progression. Functionally, the data suggested that lncRNA FGD5-AS1 positively regulated while miR-497-5p negatively modulated malignant phenotypes, including cell proliferation, viability, invasion, migration, epithelial-mesenchymal transition (EMT), and tumorigenesis in CC cells. Interestingly, the inhibiting effects of lncRNA FGD5-AS1 ablation on CC development were abrogated by both silencing miR-497-5p and upregulating PD-L1. This study found that lncRNA FGD5-AS1 sponged miR-497-5p to upregulate PD-L1, resulting in CC progression, and provided novel agents for CC diagnosis and prognosis.

## 1. Introduction

Colon cancer (CC) is the third most common malignancy, which is also the leading cause of mortality worldwide [1]. Although advances in therapy treatments had been made, poor survival and unsatisfactory prognosis remained a huge health burden for human beings [2]. Researchers agreed that uncovering the underlying mechanisms of CC pathogenesis will help to cure CC [3], and emerging evidence suggests that long noncoding RNAs (lncRNAs) are involved in regulating CC progression by serving as tumor suppressors or oncogenes [4]. For example, overexpression of LincC01082 [5] and LINC00261 [6] suppressed CC development, while lncRNA CALIC promoted malignant phenotypes in CC cells [7]. Among all the lncRNAs, we noticed that lncRNA FGD5-AS1 acted as an oncogene to facilitate the development of multiple cancers, such as colorectal cancer (CRC) [8], oral cancer [9], non-small-cell lung cancer (NSCLC) [10], and esophageal squamous cell carcinoma (ESCC) [11]. However, the role of lncRNA FGD5-AS1 in regulating CC progression is still largely unknown.

The article "Targeting the lncRNA FGD5-AS1/miR-497-5p/PD-L1 Axis Inhibits Malignant Phenotypes in Colon Cancer (CC)" was retracted in 2023. Reasons: signs of a paper mill; suspected computer-generated content; unreliable results or conclusions; concerns about the data.

There are many abnormally expressed microRNAs (miRNAs) in colon cancer, and these miRNAs can affect the biological functions of cell proliferation, invasion, and migration by regulating a variety of target genes. MicroRNAs (miRNAs) are a group of single-strand small noncoding RNAs with about 22 nucleotides [12], which are closely associated with CC development [13] and drug resistance [14]. Recent data suggested that targeting miRNAs were effective in hindering CC progression. Specifically, Mjelle et al. noticed that upregulation of miR-1273a inhibited CC development [15], and Yang et al. found that silencing of miR-122 inhibited malignant phenotypes in CC cells [16]. According to the previous publications [17], lncRNAs sponged miRNAs to regulate cancer progression in a competing endogenous RNA (ceRNA) mechanism-dependent manner [18], and Tang et al. evidenced that miR-497-5p was the downstream target of lncRNA FGD5-AS1 [19]. Interestingly, miR-497-5p served as a tumor suppressor to inhibit the development of multiple cancers, such as breast cancer (BC) [20], gastric cancer (GC) [21], and pancreatic cancer [22], and Wang et al. found that miR-497-5p mediated starvation-induced death in CC cells [23]. Nevertheless, it was still unclear whether lncRNA FGD5-AS1/miR-miR-497-5p axis regulated CC pathogenesis, making this issue meaningful and necessary.

Programmed death ligand-1 (PD-L1), also known as CD274, contributed to immune evasion and facilitated cancer progression by binding to the programmed death protein-1 (PD-1) in the membrane surface of immune cells, resulting in the dysfunctions of T lymphocytes [24]. Aside from that, recent data suggested that PD-L1 also directly promoted cancer progression, and researchers found that upregulation of PD-L1 promoted cancer cell proliferation [25], cancer stem cell (CSC) properties [26], invasion [26] and migration [27], and silencing of PD-L1 triggered apoptotic cell death in CRC [28]. Of note, PD-L1 was closely associated with the clinical prognosis in CC patients [29], and PD-L1 could be downregulated by multiple miRNAs [30]. Interestingly, Zhu et al. validated that miR-497-5p targeted the 3′ untranslated region (3′UTR) of PD-L1 mRNA for degradation in clear renal cell carcinoma (CRCC) cells [31], which rendered the possibility that lncRNA FGD5-AS1 might regulate PD-L1 through miR-497-5p in CC cells.

The article "Targeting the lncRNA FGD5-AS1/miR-497-5p/PD-L1 Axis Inhibits Malignant Phenotypes in Colon Cancer (CC)" was retracted in 2023. Reasons: signs of a paper mill; suspected computer-generated content; unreliable results or conclusions; concerns about the data.

Taken together, through *in vitro* and *in vivo* experiments, the present study managed to investigate the role of lncRNA FGD5-AS1/miR-497-5p/PD-L1 axis in regulating CC progression and uncover the potential underlying mechanisms, which will provide novel diagnostic and therapeutic agents for CC in the clinic.

## 2. Materials and Methods

### 2.1. Clinical Specimen Collection

The 50 paired cancer tissues and normal adjacent tissues were collected from colon cancer (CC) patients in the Third Affiliated Hospital of Kunming Medical University (Yunnan Cancer Hospital) from 2014 to 2018. Before surgical resection, all the participants did not accept any other therapies, such as chemotherapy and radiotherapy. The above clinical tissues were obtained and immediately stored at -70°C conditions for further analysis. All the clinical experiments were in keeping with the “Declaration of Helsinki” principle and approved by the ethics committee of The Third Affiliated Hospital of Kunming Medical University (Yunnan Cancer Hospital). In addition, the informed consent had been acquired from all the participants.

### 2.2. Cell Culture and Vector Transfection

We followed the method of Du et al. and Li et al. [5, 32]. The normal human colon epithelial cells (FHC) and colon cancer cells (SW620, HCT116, and SW480) were purchased from Obio Technology Co., Ltd., and the cells were maintained in the Dulbecco's Modified Eagle Medium (DMEM, Gibco, USA) containing 10% fetal bovine serum (FBS, Gibco, USA). All the cells were cultivated in the incubator with standard culture conditions, including a humidified atmosphere with 5% CO2 and 37°C. Next, the overexpression and downregulation vectors for lncRNA FGD5-AS1, miR-497-5p mimic and inhibitor, and PD-L1 overexpression vectors were designed and synthesized by Sangon Biotech (Shanghai, China), and the above vectors were delivered into CC cells by using the Lipofectamine 2000 reagent (Invitrogen, USA) based on the protocols provided by the manufacturer.

The article "Targeting the lncRNA FGD5-AS1/miR-497-5p/PD-L1 Axis Inhibits Malignant Phenotypes in Colon Cancer (CC)" was retracted in 2023. Reasons: signs of a paper mill; suspected computer-generated content; unreliable results or conclusions; concerns about the data.

### 2.3. Real-Time qPCR

The expression levels of lncRNA FGD5-AS1, miR-497-5p, and PD-L1 mRNA were examined by using the real-time qPCR. We followed the method of Du et al. [5]. Briefly, the total RNA was extracted by using the commercial TRIzol reagent (Invitrogen, USA), reversely transcribed by iScript cDNA synthesis kit (Bio-Rad, USA) and quantified through HiScript II Q Select RT SuperMix (Vazyme, China). The primer sequences were listed as follows: lncRNA FGD5-AS1 (Forward: 5′-GAA GGG CCG AAG AGC TCA AT-3′, Reverse: 5′-GGC TCG CAA AGT GTC TGT TG-3′), miR-497-5p (Forward: 5′-ATC CAG TGC GTG TCG TG-3′, Reverse: 5′-TGC TCA GCA GCA CAC TGT-3′), PD-L1 (Forward: 5′-CGT CTC CTC CAA ATG TGT ATC A-3′, Reverse: 5′-TGG TAA TTC TGG GAG CCA TC-3′), *β*-actin (Forward: 5′-CTC CAT CCT GGC CTC GCT GT-3′, Reverse: 5′-GCT GCT ACC TTC ACC GTT CC-3′), and U6 (Forward: 5′-GAC TAT CAT ATG CTT ACC GT-3′, Reverse: 5′-GGG CAG GAA GAG GGC CTA T-3′).

### 2.4. Western Blot Analysis

The CC cells were pretransfected with differential vectors, and the protein levels, including PD-L1, *β*-actin, N-cadherin, Vimentin, cleaved Caspase-3, and Bax were measured by using the Western blot analysis. We followed the method of Jiang et al. [33]. Briefly, the total protein was extracted by RIPA lysis buffer (Beyotime, China); protein concentrations were determined by BCA method, separated by SDS-PAGE, probed with primary and secondary antibodies, and visualized by using the ECL kit (Bio-Rad, USA). Finally, the Image J software was employed to analyze the grey values of protein bands, which were normalized to *β*-actin to reflect the relative expression levels of the proteins. All the antibodies were purchased from the Abcam Company (UK).

### 2.5. Cell Counting Kit-8 (CCK-8) Assay

We followed the method of Kawasaki et al. and Qu et al. [6, 38]. The CC cells were pretransfected with different vectors, and a commercial CCK-8 kit (MedChemExpress Co., Ltd., USA) was purchased to determine cell proliferation abilities based on the protocols provided by the producer. The HCC cells were cultured under standard conditions and incubated with CCK-8 reaction solution for 2 h at 37°C. After that, the optical density (OD) values were measured to reflect the cell proliferation of HCC cells.

### 2.6. Transwell Assay

We followed the method of Kawasaki et al. and Zhou et al. [6, 39]. The prepared CC cells were cultured in the upper compartment of the Transwell plates (Corning Co-Star, USA) in serum-free DMEM medium at the density of 2 × 10^4^ cells/well. The lower chambers were full of DMEM medium containing 10% fetal bovine serum (FBS, Gibco, USA) as chemotaxin. At 24 h postincubation, the filters were obtained and fixed with 4% paraformaldehyde and stained with 0.1% crystal violet for visualization. Finally, the cells were observed, counted, and photographed under light microscope.

The article "Targeting the lncRNA FGD5-AS1/miR-497-5p/PD-L1 Axis Inhibits Malignant Phenotypes in Colon Cancer (CC)" was retracted in 2023. Reasons: signs of a paper mill; suspected computer-generated content; unreliable results or conclusions; concerns about the data.

### 2.7. Wound Scratch Assay

We followed the method of Zhou et al. [39]. The CC cells were harvested and cultured in 6-well plates at the concentration of 3.0 × 10^4^ cells per well. After 48 h culture, a scratch was generated by using the 200 *μ*l tips, and the cell migration abilities were monitored and photographed every day under a light microscope (Thermo Fisher Scientific, USA).

### 2.8. Annexin V-FITC/PI Double Staining Assay

We followed the method of Liu et al. [40]. By using the Annexin V-FITC/PI double staining method, the cell apoptosis ratio was evaluated according to the manufacturer's instruction. Briefly, the CC cells were pretransfected with differential plasmids and subsequently incubated with Annexin V-FITC and PI reaction solution for 15 min at room temperature in darkness. After that, the flow cytometer (FCM) was used to examine the proportion of apoptotic cells.

### 2.9. Dual-Luciferase Reporter Gene System

The online staBase software (http://starbase.sysu.edu.cn/) analysis predicted the targeting sites of lncRNA FGD5-AS1, miR-497-5p, and PD-L1 mRNA, which were validated by the following dual-luciferase reporter gene system. In brief, the targeting sites in lncRNA FGD5-AS1 and 3′ UTR of PD-L1 were mutated and cloned into pGL-3 luciferase reporter vectors by a third-party company (Genescript, Nanjing, China). Next, the above vectors were cotransfected with miR-497-5p mimic and inhibitor into CC cells by using the Lipofectamine 3000 reagent (Invitrogen, USA) according to manufacturer's instruction. Finally, the relative luciferase activities were evaluated by the dual-luciferase assay system (Promega, USA).

### 2.10. *In Vivo* Animal Experiments

The male BALB/c nude mice (aged 4-6 weeks) were purchased from the Research Animal Center of Kunming Medical University, and the mice were divided into 3 groups (control group, OE-lncRNA group, and KD-lncRNA group) with 5 mice in each group and fed under the standard conditions. The CC cells were pretransfected with lncRNA FGD5-AS1 overexpression and downregulation vectors and were subcutaneously injected into the back blank of nude mice at the concentrations of 5 × 10^5^ cells per mice. At 25 days postinjection, the mice were anesthetized by intravenously injecting barbiturate at the concentration of 100 mg/kg and were subsequently sacrificed to obtain the tumors. Finally, the tumor weight was calculated to evaluate tumorigenesis of these CC cells. All the animal experiments were approved by the Ethics Committee of the Third Affiliated Hospital of Kunming Medical University (Yunnan Cancer Hospital).

The article "Targeting the lncRNA FGD5-AS1/miR-497-5p/PD-L1 Axis Inhibits Malignant Phenotypes in Colon Cancer (CC)" was retracted in 2023. Reasons: signs of a paper mill; suspected computer-generated content; unreliable results or conclusions; concerns about the data.

### 2.11. Immunohistochemistry (IHC)

We followed the method of Shan et al. [34]. The IHC assay was performed to examine the expressions and localization of Ki67 protein in mice tumor tissues. The antibody against Ki67 protein was purchased from Abcam (1 : 400, #ab245113, UK).

### 2.12. Data Analysis

All the data were collected and presented as means ± standard deviation (SD), and the data were analyzed by using the SPSS 18.0 software. Specifically, the statistical significance between two groups was analyzed by the Student's *t*-test, and one-way ANOVA analysis was used to compare the means from multiple groups. Data that were not normally distributed were analyzed with Kruskal-Wallis one-way ANOVA followed by pair-wise comparisons using Mann–Whitney *U*-tests. In addition, the Pearson correlation analysis was used to analyze the correlations of the genes in the clinical tissues. Each experiment repeated at least 3 times, and ^∗^*P* < 0.05.

## 3. Results

### 3.1. lncRNA FGD5-AS1/miR-497-5p/PD-L1 Axis was Relevant to CC Development and Prognosis

Initially, we collected 50 paired cancer tissues and their paired normal adjacent tissues from CC patients, and real-time qPCR and Western blot analysis were performed to determine the expression status of lncRNA FGD5-AS1, miR-497-5p, and PD-L1 in the above clinical tissues. As expected, we found that the expression levels of lncRNA FGD5-AS1 (Figure 1(a)) and PD-L1 mRNA (Figure 1(c)) were higher, while miR-497-5p (Figure 1(b)) was lower in CC tissues compared to the normal tissues. Consistently, 4 patients were randomly selected, and the Western blot results showed that PD-L1 was also upregulated in cancer tissues at the protein level (Figure 1(d)). Next, by conducting a Pearson correlation analysis, we found that miR-497-5p negatively correlated with lncRNA FGD5-AS1 (Figure 1(e)) and PD-L1 mRNA (Figure 1(f)), and lncRNA FGD5-AS1 was positively relevant to PD-L1 mRNA in CC tissues (Figure 1(g)). Additionally, we selected the normal human colon epithelial cells (FHC) and CC cells (SW620, HCT116, and SW480) for further cellular analysis, and the results evidenced that lncRNA FGD5-AS1 (Figure 1(h)) and PD-L1 (Figures 1(j) and 1(k)) were upregulated, while miR-497-5p was downregulated in CC cells (Figure 1(i)), in contrast with the FHC cells.

### 3.2. lncRNA FGD5-AS1 Positively Regulated CC Progression *In Vitro* and *In Vivo*

The overexpression and downregulation vectors for lncRNA FGD5-AS1 were delivered into CC cells (Figure 2(a)), and further experiments validated that lncRNA FGD5-AS1 functioned as an oncogene to promote CC development. Specifically, by conducting the CCK-8 assay, we validated that lncRNA FGD5-AS1 overexpression promoted cell proliferation in CC cells, but silencing of lncRNA FGD5-AS1 had opposite effects (Figures 2(b)–2(d)). Next, by performing the Transwell assay and wound scratch assay, we found that lncRNA FGD5-AS1 also positively regulated cell invasion (Figure 2(e)) and migration (Figure 2(f)) in CC cells. Furthermore, the Annexin V-FITC/PI double staining assay was performed to examine cell apoptosis, and we found that knock-down of lncRNA FGD5-AS1 triggered apoptotic cell death in CC cells (Figure 2(g)). Finally, the CC cells with lncRNA FGD5-AS1 overexpression and deficiency were employed to establish xenograft tumor-bearing mice models *in vivo*, and we found that deficiency of lncRNA FGD5-AS1 decreased tumor weight to inhibit tumorigenesis in CC cells, while lncRNA FGD5-AS1 overexpression had opposite effects (Figures S1A, S2A, and S3A). Consistently, the immunohistochemistry (IHC) assay results showed that lncRNA FGD5-AS1 positively regulated Ki67 protein levels in mice tumor tissues (Figures S1B, S2B, and S3B).

The article "Targeting the lncRNA FGD5-AS1/miR-497-5p/PD-L1 Axis Inhibits Malignant Phenotypes in Colon Cancer (CC)" was retracted in 2023. Reasons: signs of a paper mill; suspected computer-generated content; unreliable results or conclusions; concerns about the data.

### 3.3. MiR-497-5p Acted as a Tumor Suppressor in CC Development

Since miR-497-5p was downregulated in CC tissues and cell lines, we next investigated the regulating mechanisms of miR-497-5p in CC pathogenesis by transfecting the miR-497-5p mimic and inhibitor into CC cells (Figure 3(a)). As shown in Figures 3(b)–3(d), the CCK-8 assay results indicated that overexpression of miR-497-5p inhibited cell proliferation, which were promoted by silencing miR-497-5p in CC cells. Next, we found that miR-497-5p overexpression inhibited cell invasion (Figure 3(e)) and migration (Figure 3(f)) abilities in CC cells, while silencing of miR-497-5p promoted cell mobility (Figures 3(e) and 3(f)). Similarly, the Western blot analysis results suggested that miR-497-5p negatively regulated N-cadherin and Vimentin to inhibit EMT in CC cells (Figure S4A-C). Also, we found that upregulation of miR-497-5p promoted cell apoptosis in CC cells (Figure 3(g)), and the Western blot analysis results evidenced that miR-497-5p overexpression increased cleaved caspase-3 and Bax to induce cell apoptosis (Figure S5A-C) and inhibited cyclin D1 and CDK2 to hinder cell cycle in CC cells (Figure S6A-C).

### 3.4. lncRNA FGD5-AS1 Promoted PD-L1 Expressions in CC Cells by Targeting miR-497-5p

The online starBase software (http://starbase.sysu.edu.cn/) and miRDB database (http://mirdb.org/) indicated that miR-497-5p potentially targeted lncRNA FGD5-AS1 (Figure 4(a)) and 3′ untranslated region (UTR) of PD-L1 mRNA (Figure 4(e)), indicating that there might exist regulatory mechanisms among lncRNA FGD5-AS1, miR-497-5p, and PD-L1. The above hypothesis was validated by the following dual-luciferase reporter gene system assay, which showed that the luciferase activity were decreased by miR-497-5p mimic, and increased by miR-497-5p inhibitor in the CC cells cotransfected with Wt-FGD5-AS1 (Figures 4(b)–4(d)) and Wt-PD-L1 (Figures 4(f)–4(h)), instead of their mutant counterparts. Furthermore, by conducting the real-time qPCR and Western blot analysis, we found that lncRNA FGD5-AS1 upregulated PD-L1 in CC cells by sponging miR-497-5p. Specifically, miR-497-5p decreased the expression levels of PD-L1 at both transcriptional (Figure 4(i)) and translated levels (Figure 4(j)). In addition, we found that upregulation of lncRNA FGD5-AS1 promoted PD-L1 expressions, which were reversed by overexpressing miR-497-5p (Figures 4(k) and 4(l)).

The article "Targeting the lncRNA FGD5-AS1/miR-497-5p/PD-L1 Axis Inhibits Malignant Phenotypes in Colon Cancer (CC)" was retracted in 2023. Reasons: signs of a paper mill; suspected computer-generated content; unreliable results or conclusions; concerns about the data.

### 3.5. Knock-Down of lncRNA FGD5-AS1 Hampered CC Development by Targeting miR-497-5p and PD-L1

Finally, the underlying mechanisms of lncRNA FGD-AS1/miR-497-5p/PD-L1 axis regulated CC progression were investigated. As shown in Figures 5(a)–5(c), we found that the inhibiting effects of lncRNA FGD5-AS1 ablation on cell proliferation in CC cells were abrogated by downregulating miR-497-5p and upregulating PD-L1. Similarly, the Transwell assay and wound scratch assay results suggested that silencing of lncRNA FGD5-AS1 inhibited cell invasion and migration in CC cells, which were reversed by knocking down miR-497-5p and overexpressing PD-L1 (Figures 5(d) and 5(e)). Also, knock-down of lncRNA FGD5-AS1 decreased the expression levels of N-cadherin and Vimentin to inhibit EMT by downregulating miR-497-5p and upregulating PD-L1 in CC cells (Figure S7A-C). In addition, by performing the Annexin V-FITC/PI double staining assay, we found that knock-down of lncRNA FGD5-AS1 triggered apoptotic cell death in CC cells, which were rescued by silencing miR-497-5p and upregulating PD-L1 (Figure 5(f)).

## 4. Discussion

Recently, targeting lncRNAs-miRNAs-mRNAs ceRNA networks proved to be an effective strategy to slow down the development of multiple cancers [35], and the present study identified a novel lncRNA FGD5-AS1/miR-497-5p/PD-L1 axis that played an important role in regulating colon cancer (CC) progression. Mechanistically, we found that lncRNA FGD5-AS1 tended to be enriched in CC tissues and cells compared to their normal counterparts. Further gain- and loss-function experiments validated that overexpression of lncRNA FGD5-AS1 promoted the malignant phenotypes, including cell proliferation, invasion, migration, and tumorigenesis in CC cells *in vitro* and *in vivo*, while silencing of lncRNA FGD5-AS1 had opposite effects on the above cell functions, suggesting that lncRNA FGD5-AS1 acted as an oncogene to promote CC development, which was in accordance with the previous publications in other types of cancer [36].

The article "Targeting the lncRNA FGD5-AS1/miR-497-5p/PD-L1 Axis Inhibits Malignant Phenotypes in Colon Cancer (CC)" was retracted in 2023. Reasons: signs of a paper mill; suspected computer-generated content; unreliable results or conclusions; concerns about the data.

Given the fact that miR-497-5p served as a tumor suppressor to inhibit the development of multiple cancers [37], we proved that upregulation of miR-497-5p also hindered the development of CC. Specifically, the expression levels of miR-497-5p were decreased in CC tissues and cells. Also, the miR-497-5p was overexpressed and silenced in the CC cells, and the results showed that upregulation of miR-497-5p inhibited cell proliferation, migration, and epithelial-mesenchymal transition (EMT), and promoted cell apoptosis in CC cells, but miR-497-5p overexpression promoted the development of CC *in vitro*. Consistently, further experiments validated that overexpression of miR-497-5p increased the expression levels of proapoptosis-associated proteins (cleaved Caspase-3 and Bax), but inhibited proliferation associated proteins (Cyclin D1 and CDK2) in CC cells. The above results suggested that miR-497-5p inhibited CC pathogenesis, which was supported by the previous work [37]. In addition, the levels of miR-497-5p negatively correlated with lncRNA FGD5-AS1, and Tang et al. evidenced that miR-497-5p potentially bound to lncRNA FGD5-AS1 [19]. Based on this, we validated that lncRNA FGD5-AS1 sponged miR-497-5p to facilitate CC progression.

Recent data agreed that programmed death ligand-1 (PD-L1) participated in regulating cancer progression through immune evasion [24]. Besides that, researchers found that PD-L1 acted as an oncogene to accelerate cancer development by directly regulating malignant phenotypes [38]. By conducting the clinical experiments, we validated that PD-L1 tended to be enriched in CC tissues and cells, instead of their normal counterparts. In addition, Zhu et al. validated that PD-L1 was the downstream target of miR-497-5p in clear renal cell carcinoma (CRCC) cells [31], and lncRNA FGD5-AS1 acted as a RNA sponge for miR-497-5p [19]. Also, our clinical data suggested that PD-L1 mRNA was positively relevant to lncRNA FGD5-AS1, while negatively correlated with miR-497-5p in CC tissues. Based on this, we proved that lncRNA FGD5-AS1 sponged miR-497-5p to upregulate PD-L1 in CC cells. Furthermore, upregulation of PD-L1 abrogated the inhibiting effects of lncRNA FGD5-AS1 ablation on CC development, suggesting that silencing of lncRNA FGD5-AS1 hindered CC progression through downregulating PD-L1.

## 5. Conclusions

Collectively, we proved that silencing of lncRNA FGD5-AS1 upregulated PD-L1 through sponging miR-497-5p to inhibit malignant phenotypes, including cell proliferation, viability, invasion, migration, and EMT in CC cells *in vitro* and *in vivo*. The present study provided novel biomarkers for CC diagnosis and treatment and broadened our knowledge in this field.

The article "Targeting the lncRNA FGD5-AS1/miR-497-5p/PD-L1 Axis Inhibits Malignant Phenotypes in Colon Cancer (CC)" was retracted in 2023. Reasons: signs of a paper mill; suspected computer-generated content; unreliable results or conclusions; concerns about the data.

## Figures and Tables

**Figure 1:** The expression levels of lncRNA FGD5-AS1, miR-497-5p, and PD-L1 in CC tissues and cells. Real-time qPCR was used to examine the expression levels of (a) lncRNA FGD5-AS1, (b) miR-497-5p, and (c) PD-L1 mRNA in CC tissues and normal adjacent tissues. (d) Western blot analysis was conducted to determine the protein levels of PD-L1 in CC tissues. (e–g) Pearson correlation analysis was conducted to determine the correlations of lncRNA FGD5-AS1, miR-497-5p, and PD-L1 mRNA in CC tissues. The expression levels of (h) lncRNA FGD5-AS1, (i) miR-497-5p, and (j) PD-L1 mRNA in CC cells. (k) Western blot was used to detect the protein levels of PD-L1 in CC cells. Each experiment repeated at least 3 times, and “^∗^” represented *P* < 0.05.

**Figure 2:** lncRNA FGD5-AS1 promoted cancer progression in CC. (a) The overexpression and downregulation vectors for lncRNA FGD5-AS1 were delivered into CC cells. (b–d) CCK-8 assay was used to determine cell proliferation in CC cells. (e) Transwell assay was employed to evaluate cell invasion. (f) Wound scratch assay was performed to determine cell migration. (g) Cell apoptosis ratio was determined by using the Annexin V-FITC/PI double staining assay. Each experiment repeated at least 3 times, and “^∗^” represented *P* < 0.05.

**Figure 3:** Upregulation of miR-497-5p inhibited malignant phenotypes in CC cells. (a) The miR-497-5p mimic and inhibitor were used to overexpress and silence miR-497-5p in CC cells. (b–d) CCK-8 assay was conducted to measure cell proliferation. (e) Cell invasion was determined by Transwell assay. (f) Wound scratch assay was used to determine cell migration. (g) Annexin V-FITC/PI double staining assay was used to determine cell apoptosis. Each experiment repeated at least 3 times, and “^∗^” represented *P* < 0.05.

**Figure 4:** lncRNA FGD5-AS1 sponged miR-497-5p to upregulate PD-L1 in CC cells. The online starBase software (http://starbase.sysu.edu.cn/) was used to predict the binding sites of miR-497-5p with (a) lncRNA FGD5-AS1 and (e) 3′UTR of PD-L1 mRNA. The binding sites of miR-497-5p with (b–d) lncRNA FGD5-AS1 and (f–h) 3′UTR of PD-L1 mRNA were validated by using the dual-luciferase reporter gene system assay. MiR-497-5p negatively regulated PD-L1 at (i) transcriptional and (j) translated levels. (k, l) Upregulation of lncRNA FGD5-AS1 promoted PD-L1 expressions through downregulating miR-497-5p. Each experiment repeated at least 3 times, and “^∗^” represented *P* < 0.05.

The article "Targeting the lncRNA FGD5-AS1/miR-497-5p/PD-L1 Axis Inhibits Malignant Phenotypes in Colon Cancer (CC)" was retracted in 2023. Reasons: signs of a paper mill; suspected computer-generated content; unreliable results or conclusions; concerns about the data.

**Figure 5:** Knock-down of lncRNA FGD5-AS1 inhibited CC progression through targeting miR-497-5p/PD-L1 axis. (a–c) CCK-8 assay was used to examine cell proliferation in CC cells. (d) Transwell assay and (e) wound scratch assay were conducted to measure cell mobility in CC cells. (f) Annexin V-FITC/PI double staining assay was employed to measure cell apoptosis in CC cells. Each experiment repeated at least 3 times, and “^∗^” represented *P* < 0.05.

## Data Availability

No data were used to support this study.

## Supplementary Materials

Supplementary Materials Supplementary Figure 1: lncRNA FGD5-AS1 positively regulated CC progression *in vivo*. (A) Observation of tumor size and weight in mouse xenograft tumor models established by SW620 cells. (B) Detection of Ki67 protein level in mouse tumor tissue by immunohistochemistry (IHC). Each experiment repeated at least 5 times, and “^∗^” represented *P* < 0.05. Supplementary Figure 2: lncRNA FGD5-AS1 positively regulated CC progression *in vivo*. (A) Observation of tumor size and weight in mouse xenograft tumor models established by HCT116 cells. (B) Detection of Ki67 protein level in mouse tumor tissue by immunohistochemistry (IHC). Each experiment repeated at least 5 times, and “^∗^” represented *P* < 0.05. Supplementary Figure 3: lncRNA FGD5-AS1 positively regulated CC progression *in vivo*. (A) Observation of tumor size and weight in mouse xenograft tumor models established by SW480 cells. (B) Detection of Ki67 protein level in mouse tumor tissue by immunohistochemistry (IHC). Each experiment repeated at least 5 times, and “^∗^” represented *P* < 0.05. Supplementary Figure 4: miR-497-5p acted as a tumor suppressor in CC development. (A) Western blot was used to detect the expression of EMT-related proteins N-cadherin and Vimentin in SW620 cells. (B) Western blot was used to detect the expression of EMT-related proteins N-cadherin and Vimentin in HCT116 cells. (C) Western blot was used to detect the expression of EMT-related proteins N-cadherin and Vimentin in SW480 cells. Each experiment repeated at least 3 times, and “^∗^” represented *P* < 0.05. Supplementary Figure 5: miR-497-5p acted as a tumor suppressor in CC development. (A) Western blot was used to detect the expression of apoptosis-related proteins caspase-3 and Bax in SW620 cells. (B) Western blot was used to detect the expression of apoptosis-related proteins caspase-3 and Bax in HCT116 cells. (C) Western blot was used to detect the expression of apoptosis-related proteins caspase-3 and Bax in SW480 cells. Each experiment repeated at least 3 times, and “^∗^” represented *P* < 0.05. Supplementary Figure 6: miR-497-5p acted as a tumor suppressor in CC development. (A) Western blot was used to detect the expression of cell cycle-related proteins Cyclin D1 and CDK2 in SW620 cells. (B) Western blot was used to detect the expression of cell cycle-related proteins Cyclin D1 and CDK2 in HCT116 cells. (C) Western blot was used to detect the expression of cell cycle-related proteins Cyclin D1 and CDK2 in SW480 cells. Each experiment repeated at least 3 times, and “^∗^” represented *P* < 0.05. Supplementary Figure 7: knock-down of lncRNA FGD5-AS1 inhibited CC progression through targeting miR-497-5p/PD-L1 axis. (A) Western blot was used to detect the expression of EMT-related proteins N-cadherin and Vimentin in SW620 cells. (B) Western blot was used to detect the expression of EMT-related proteins N-cadherin and Vimentin in HCT116 cells. (C) Western blot was used to detect the expression of EMT-related proteins N-cadherin and Vimentin in SW480 cells. Each experiment repeated at least 3 times, and “^∗^” represented *P* < 0.05.
